The article "Osthole resensitizes CD133+ hepatocellular carcinoma cells to cisplatin treatment via PTEN/AKT pathway" was published in 2020. Journal: Aging (Albany NY).

# Osthole resensitizes CD133^+^ hepatocellular carcinoma cells to cisplatin treatment via PTEN/AKT pathway

**DOI:** 10.18632/aging.103484

**Published:** 2020-07-16

**Authors:** Junfeng Ye, Di Sun, Ying Yu, Jinhai Yu

**Affiliations:** 1 Department of Hepato-Biliary-Pancreatic Surgery, First Hospital Jilin University, Changchun 130021, Jilin Province, China; 2 Department of Colorectal and Anal Surgery, First Hospital Jilin University, Changchun 130021, Jilin Province,130021, China; 3 Department of Gastrointestinal Surgery, First Hospital Jilin University, Changchun 130021, Jilin Province, China

**Keywords:** osthole, PTEN, AKT, Bcl-2, cisplatin

## Abstract

The population of CD133 positive cancer cells has been reported to be responsible for drug resistance of hepatocellular carcinoma (HCC). However, the potential molecular mechanism by which CD133^+^ HCC cells develop drug resistance is still unclear. In this study, we found that CD133^+^ HepG2 and Huh7 cells were resistant to cisplatin treatment, compared to the CD133^-^ HepG2 and Huh7 cells. However, treatment with osthole, a natural coumarin isolated from umbelliferae plant monomers, was found to resensitize CD133^+^ HepG2 and Huh7 cells to cisplatin treatment. In the mechanism research, we found that treatment with osthole increased the expression of PTEN. As a result, osthole inhibited the phosphorylation of AKT and Bad to decrease the amount of free Bcl-2 in CD133^+^ HepG2 and Huh7 cells. Finally, cisplatin-induced mitochondrial apoptosis was expanded. In conclusion, combination treatment with osthole can resensitize CD133^+^ HCC cells to cisplatin treatment via the PTEN/AKT pathway.

## INTRODUCTION

Hepatocellular carcinoma (HCC) is one of the most common and lethal human malignant cancers worldwide [1, 2]. Although surgery treatment is the most effective treatment strategy for the early stage of HCC, tumors in many HCC patients are unresectable because they are usually diagnosed in an advanced stage. For these patients, the systematic chemotherapy and immunotherapy are irreplaceable and valuable [3–6]. Unfortunately, cancer cells usually develop mechanisms to acquire the resistance against anti-tumor drugs [7, 8]. Recently, studies demonstrate that drug resistance is partially induced by a population of CD133 positive cells in some cancers including HCC [9–11].

CD133 is a glycoprotein on cell surface. Previous studies have indicated that cancer cells which express CD133 exhibit “stem-like”, and thus they are called “cancer stem cells” [12–14]. These CD133 positive cancer cells have high self-renewal capacity and multilineage differentiation potential. They are important for tumor formation and development [15, 16]. Furthermore, studies indicate that CD133 positive cells are responsible for the high resistance to chemotherapeutic drugs [17, 18]. This population of cancer cells may represent a novel target for improving the chemotherapy.

Previous studies have proved that some natural plants are a significant source of potential drugs against cancer. Among these natural drugs, osthole has been reported to inhibit the growth of some cancers [19–21]. Osthole is a natural coumarin that is isolated from *Cnidium monnieri*. Its chemical formula is C_15_H_16_O_3_. Studies indicate that osthole exerts a wide variety of biological effects including anti-seizure, anti-osteoporosis and anti-inflammation [22–24]. More importantly, studies have found that osthole can partially inhibit the epithelial-mesenchymal transition process and induce apoptosis or cell cycle arrest in some cancers [25, 26]. However, little is known regarding to the effect of osthole on the chemoresistance of HCC. The aim of this study is to explore the effect of osthole on cisplatin treatment against CD133^+^ HCC cells which are chemoresistant.

## RESULTS

### CD133 positive HCC cells were resistant to cisplatin

We first separated CD133 positive and negative population in Huh7 and HepG2 cell lines, the purity of these two populations was detected by flow cytometry (Figure 1A). Under the treatment of cisplatin with equal concentrations, we found significant resistance in CD133^+^ Huh7 and HepG2 cells compared to the CD133^-^ Huh7 and HepG2 cells (*P*<0.05) (Figure 1B). We confirmed that IC50 of cisplatin to CD133^+^ Huh7 cells was 4.64 fold higher than that to CD133^-^ Huh7 cells (*P*<0.05). Meanwhile, IC50 of cisplatin to CD133^+^ HepG2 cells was 5.32 fold higher than that to CD133^-^ HepG2 cells (*P*<0.05) (Figure 1C). We demonstrated that CD133 positive HCC cells were resistant to cisplatin.

**Figure 1:** **Cisplatin resistance of CD133^+^ HCC cells.** (**A**) Purity of sorted CD133^+^ and CD133^-^ Huh7 and HepG2 cells was tested by flow cytometry. (**B**) Sensitization of CD133^+^ and CD133^-^ Huh7 and HepG2 cells to different concentrations of cisplatin (0~30 μM). *P<0.05. (**C**) IC50 of cisplatin to CD133^+^ and CD133^-^ Huh7 and HepG2 cells. ^#^*P*<0.05 *vs.* CD133^-^ population.

### Downregulation of PTEN is responsible for the cisplatin resistance of CD133^+^ HCC cells

Results of western blot analysis showed that expression of PTEN was significantly lower in CD133^+^ Huh7 and HepG2 cells compared to the CD133^-^ Huh7 and HepG2 cells (*P*<0.05) (Figure 2A). To explore whether the CD133 positive HCC cells exhibited significant cisplatin resistance was associated with downregulation of PTEN, we compulsively expressed the PTEN in CD133^+^ Huh7 and HepG2 cells by using PTEN eukaryotic expression plasmid (Figure 2B). We then found that recovery of PTEN expression in CD133^+^ Huh7 and HepG2 cells increased their sensitivity to cisplatin treatment (*P*<0.05) (Figure 2C). On the other hand, we performed a loss-of-function test on PTEN by using PTEN specific siRNA in CD133^-^ Huh7 and HepG2 cells (Figure 2D). We then found that knockdown of PTEN induced significant cisplatin resistance in CD133^-^ Huh7 and HepG2 cells (*P*<0.05) (Figure 2E). These data indicated that PTEN expression partially determined the sensitivity of cisplatin to HCC. Downregulation of PTEN is responsible for the cisplatin resistance of CD133 positive HCC cells.

**Figure 2:** **Effect of PTEN on regulating the cisplatin sensitivity of CD133^+^ and CD133^-^ HCC cells.** (**A**) expression of PTEN in CD133^+^ and CD133^-^ Huh7 and HepG2 cells. ^&^*P*<0.05 *vs.* CD133^-^ Huh7 cells, ^#^*P*<0.05 *vs.* CD133^-^ HepG2 cells. (**B**) Transfection with PTEN plasmid increased the expression of PTEN in CD133^+^ Huh7 and HepG2 cells. *P<0.05. (**C**) Transfection with PTEN plasmid increased the sensitivity of CD133^+^ Huh7 and HepG2 cells to cisplatin (5 μM) treatment. *P<0.05. (**D**) Transfection with PTEN siRNA decreased the expression of PTEN in CD133^-^ Huh7 and HepG2 cells. *P<0.05. (**E**) Transfection with PTEN siRNA decreased the sensitivity of CD133^-^ Huh7 and HepG2 cells to cisplatin (5 μM) treatment. *P<0.05.

### Osthole decreased the cisplatin resistance of CD133 positive HCC cells

To explore whether the osthole affected the chemoresistance of CD133 positive HCC cells, we co-treated the CD133^+^ Huh7 and HepG2 cells with cisplatin and osthole. Comparing to the cisplatin single treatment groups, combination treatment groups with cisplatin and osthole showed lower cell viability (*P*<0.05) (Figure 3A). We confirmed that osthole decreased the IC50 of cisplatin by 84.3% to CD133^+^ Huh7 cells and 80.5% to CD133^+^ HepG2 cells (*P*<0.05) (Figure 3B). Furthermore, we calculated that combination index (CI) with cisplatin and osthole was greater than 1.15 in CD133^+^ Huh7 cells (Table 1) and CD133^+^ HepG2 cells (Table 2). These data demonstrated that osthole exhibited synergistic effect on cisplatin. On the other hand, we tested the effect of osthole on the CD133^-^ HCC cells. We found that osthole decreased the IC50 of cisplatin by 47.5% to CD133^-^ Huh7 cells and 40.7% to CD133^-^ HepG2 cells (*P*<0.05) (Figure 3C). These data indicated that CD133^+^ HCC cells are more sensitive to osthole than the CD133^-^ HCC cells. Treatment with osthole can decrease the cisplatin resistance of CD133 positive HCC cells.

**Figure 3:** **Osthole partially reversed the cisplatin resistance of CD133^+^ HCC cells.** (**A**) Combination treatment with osthole (10 μmol/L) increased the cytotoxicity of cisplatin (0~30 μM) against CD133^+^ Huh7 and HepG2 cells. *P<0.05. (**B**) Osthole (10 μmol/L) decreased the IC50 of cisplatin to CD133^+^ Huh7 and HepG2 cells. ^#^*P*<0.05 *vs.* Control group. (**C**) Effect of osthole (10 μmol/L) on decreasing the IC50 of cisplatin to CD133^-^ Huh7 and HepG2 cells. ^#^*P*<0.05 *vs.* Control group.

**Table 1:** Combination index (CI) with cisplatin and osthole in CD133^+^ Huh7.

**Cisplatin single treatment**		**Osthole single treatment**		**Combination treatment**	**Combination index (CI)**
**Concentration (μM)**	**Inhibitory rate (%)**	**Concentration (μM)**	**Inhibitory rate (%)**	**Inhibitory rate (%)**	
1	2.1	2	3.8	20.4	3.51
2	4.4	4	4.9	32.6	3.59
5	8.7	10	6.3	55.2	3.82
10	16.5	20	8.8	62.8	2.63
15	22.7	30	12.6	67.6	2.08
20	28.8	40	14.5	73.4	1.88
30	37.9	60	16.3	79.5	1.66

**Table 2:** Combination index (CI) with cisplatin and osthole in CD133^+^ HepG2.

**Cisplatin single treatment**		**Osthole single treatment**		**Combination treatment**	**Combination index (CI)**
**Concentration (μM)**	**Inhibitory rate (%)**	**Concentration (μM)**	**Inhibitory rate (%)**	**Inhibitory rate (%)**	
1	2.4	2	4.0	18.5	2.93
2	5.2	4	4.6	33.2	3.47
5	10.5	10	6.8	59.3	3.58
10	19.4	20	9.4	66.3	2.46
15	26.2	30	14.1	71.7	1.96
20	35.9	40	15.8	77.2	1.68
30	44.7	60	18.4	82.6	1.51

### Osthole partially reversed the cisplatin resistance of CD133 positive HCC cells through upregulation of PTEN

Results of qRT-PCR and western blot analysis showed that osthole treatment can increase the expression of PTEN at the mRNA level (Figure 4A) and the protein level (Figure 4B) in CD133^+^ Huh7 and HepG2 cells. To investigate whether the osthole resensitized CD133 positive HCC cells to cisplatin was dependent on the upregulation of PTEN, we knocked down the PTEN in CD133^+^ Huh7 and HepG2 cells by using PTEN siRNA (Figure 4B). Results of CCK-8 assays showed that treatment with osthole significantly increased the cytotoxicity of cisplatin against CD133^+^ Huh7 and HepG2 cells (*P*<0.05). However, knockdown of PTEN abolished the effect of osthole (*P*<0.05) (Figure 4C). Moreover, results of flow cytometry showed that CD133^+^ Huh7 and HepG2 cells were resistant to cisplatin-induced apoptosis. However, osthole resensitized the cisplatin-induced apoptosis (*P*<0.05). On the other hand, transfection with PTEN siRNA inhibited the apoptosis induced by the combination treatment with cisplatin and osthole (*P*<0.05) (Figure 4D). Taken together, these results indicated that osthole partially reversed the resistance of CD133 positive HCC cells to cisplatin-induced apoptosis through upregulation of PTEN.

**Figure 4:** **Osthole partially reversed the cisplatin resistance of CD133^+^ HCC cells through the PTEN pathway.** (**A**) QRT-PCR analysis was used to test the effect of osthole (10 μmol/L) on changing the expression of PTEN at the mRNA level. ^#^*P*<0.05 *vs.* control group, ^&^*P*<0.05 *vs.* cisplatin group. (**B**) Western blot analysis was used to evaluate the effect of osthole (10 μmol/L) and PTEN siRNA on affecting the expression of PTEN at the protein level. (**C**) Transfection with PTEN siRNA increased the cell viability of CD133^+^ Huh7 and HepG2 cells which were co-treated with osthole (10 μmol/L) and cisplatin (5 μmol/L). ^#^*P*<0.05 *vs.* cisplatin+control siRNA group, ^&^*P*<0.05 *vs.* cisplatin+osthole+control siRNA group. (**D**) Transfection with PTEN siRNA decreased the apoptotic rate of CD133^+^ Huh7 and HepG2 cells which were co-treated with osthole (10 μmol/L) and cisplatin (5 μmol/L). ^#^*P*<0.05 *vs.* cisplatin+control siRNA group, ^&^*P*<0.05 *vs.* cisplatin+osthole+control siRNA group.

### Osthole sensitized the cisplatin-induced apoptosis through the PTEN/AKT/Bad/Bcl-2 pathway

Previous study has reported that inhibition of PTEN leads to phosphorylation of AKT [27]. We thus evaluated the role of AKT in CD133^+^ HCC cells. Results of western blot analysis showed that osthole treatment can reduce the level of phosphorylated AKT (p-AKT) no matter whether the CD133^+^ Huh7 and HepG2 cells were treated with cisplatin or not. However, knockdown of PTEN was found to abolish the effect of osthole on inhibiting the AKT phosphorylation (Figure 5A). It indicated that osthole treatment reduced the phosphorylation of AKT through the PTEN pathway. Bad, a pro-apoptotic protein, is one of the substrates for AKT [28]. We next found that osthole treatment inhibited the phosphorylation of Bad through increase of PTEN expression (Figure 5A). As osthole decreased the phosphorylation of Bad, results of immunoprecipitation (IP) showed that osthole treatment enhanced the heterodimerization of Bad and Bcl-2 in CD133^+^ Huh7 and HepG2 cells (Figure 5B). As a result, osthole inactivated the Bcl-2 which is the key anti-apoptotic protein through the PTEN/AKT/Bad pathway. To evaluate the function of mitochondria, we next tested the mitochondrial membrane potential (ΔΨ_m_) and cytosolic cytochrome c in CD133^+^ Huh7 and HepG2 cells. Results of flow cytometry showed that combination treatment with osthole enhanced the effect of cisplatin on reducing the ΔΨ_m_ of CD133^+^ Huh7 and HepG2 cells (Figure 5C). Furthermore, we found the obvious release of cytochrome c in osthole and cisplatin co-treated CD133^+^ Huh7 and HepG2 cells (Figure 5D). However, transfection with PTEN siRNA abolished the effect of osthole. As the results of mitochondria dysfunction, caspase-9 and caspase-3 were activated in CD133^+^ Huh7 and HepG2 cells which were co-treated with osthole and cisplatin (Figure 5E). Taken together, we demonstrated that osthole can sensitize the cisplatin-induced apoptosis through the PTEN/AKT/Bad/Bcl-2 pathway in CD133 positive HCC cells.

**Figure 5:** **osthole enhanced the cisplatin-induced apoptosis through the PTEN/AKT/Bad/Bcl-2 pathway in CD133^+^ HCC cells.** (**A**) Effect of osthole (10 μmol/L) and PTEN siRNA on affecting the phosphorylation of AKT and Bad in CD133^+^ Huh7 and HepG2 cells. (**B**) Effect of osthole (10 μmol/L) and PTEN siRNA on affecting the interaction with Bad and Bcl-2 in CD133^+^ Huh7 and HepG2 cells. (**C**) Osthole (10 μmol/L) enhanced the effect of cisplatin (5 μmol/L) on reducing the mitochondrial membrane potential (ΔΨ_m_) of CD133^+^ Huh7 and HepG2 cells. (**D**) Osthole (10 μmol/L) increased the cytosolic cytochrome c in CD133^+^ Huh7 and HepG2 cells which were treated with cisplatin (5 μmol/L). (**E**) Osthole (10 μmol/L) increased the apoptotic rate of CD133^+^ Huh7 and HepG2 cells which were treated with cisplatin (5 μmol/L).

### Osthole attenuated the cisplatin resistance of CD133 positive HCC in vivo

To test the effect of osthole on CD133 positive HCC in vivo, we inoculated the CD133^+^ Huh7 cells into the nude mice before treatment with osthole and cisplatin. We found that the growth of tumors which were co-treated with osthole and cisplatin was obviously slower than the tumors treated with single cisplatin or osthole (Figure 6A). After euthanasia of nude mice followed by separation of tumor tissues, we observed that the tumors which were co-treated with osthole and cisplatin were smaller and lighter than the tumors treated with single cisplatin or osthole (*P*<0.05) (Figure 6B, 6C). On the other hand, results of western blot analysis showed obvious upregulation of PTEN expression in osthole-treated tumors (Figure 6D). Furthermore, we found that osthole enhanced the effect of cisplatin on triggering the caspase-9 and caspase-3 which were the apoptosis markers (Figure 6E). Taken together, These data demonstrated that osthole treatment can attenuate the cisplatin resistance of CD133 positive HCC in vivo.

**Figure 6:** **Osthole attenuated the cisplatin resistance of CD133 positive HCC in vivo.** (**A**) Growth curve of CD133^+^ Huh7 originated tumors on nude mice which were treated with cisplatin (8 mg/kg) and osthole (20 mg/kg) twice a week. (**B**) Separated tumor tissues from nude mice after euthanasia. (**C**) The final weight of separated tumor tissues from nude mice after euthanasia. *P<0.05 *vs.* osthole treatment group, ^#^*P*<0.05 *vs.* cisplatin treatment group. (**D**) Expression of PTEN in purified tumor tissues was tested by western blot analysis. (**E**) Activation of caspase-9 and caspase-3 in purified tumor tissues was tested by western blot analysis.

## DISCUSSION

Cisplatin is a platinum-based antineoplastic drug that cross-links with DNA of cancer cells. Subsequently, cisplatin inhibits DNA replication and induces apoptosis of cancer cells [29, 30]. As a broad-spectrum antineoplastic drug, cisplatin is commonly used for the treatment of multiple malignant cancers including HCC [31–33]. However, the population of CD133 positive HCC cells showed significant resistance to cisplatin and is responsible for the failure of cisplatin treatment [34]. To improve the curative effect of cisplatin on HCC, CD133 positive cells are important targets. In the present study, we separated the CD133 positive and CD133 negative cells from the HCC cell lines Huh7 and HepG2. We then found that CD133 positive HCC cells exhibited significant cisplatin resistance compared to the CD133 negative HCC cells. It is urgent to overcome the drug resistance of CD133 positive HCC cells.

Studies have reported that multiple natural drugs can be used as sensitizers in chemotherapy. For instance, imperatorin, a linear furanocoumarin compound extracted from the root of *Angelica dahurica*, has been reported to decrease the cisplatin resistance through suppression of MCL-1 [35]; Quercetin, a flavonoid that widely distributes in plant-based foods, has been found to reverse the resistance of prostate cancer to doxorubicin-based therapy [36]; Resveratrol, a natural polyphenol compound, has been proved to restore the sensitivity of glioma cells to temozolamide through inhibiting the activation of Wnt signaling pathway [37]. As one kind of natural drug, osthole has some anti-tumor activity with low toxicity and little side effects. Furthermore, we found the adjuvant effect of osthole on CD133 positive HCC cells in this study. Our results showed that combination index (CI) with cisplatin and osthole on CD133 positive HCC cells was greater than 1.15. These results indicated that osthole can be used as a sensitizer and had synergistic effect on cisplatin. We proved that treatment with osthole can partially reverse the cisplatin resistance of CD133 positive HCC cells.

Phosphatase and tensin homologue (PTEN) has been reported to act as an important tumor suppressor, because it inhibits tumorigenesis and cancer development. Loss of PTEN accumulates the phosphatidylinositol 3, 4, 5-trisphosphate (PIP3) and thus leads to phosphorylation of AKT. As a result, cells develop uncontrolled cell cycle [38, 39]. In this study, we indicated that the drug resistance of CD133 positive HCC cells was associated with the dysfunction of PTEN/AKT-signaling pathway. Furthermore, our results showed that the CD133 positive HCC cells were more sensitive to osthole than the CD133 negative HCC cells. We explained that the synergistic effect of osthole on cisplatin was dependent on the increase of PTEN expression, and the osthole obviously corrected the absence of PTEN in CD133 positive HCC cells.

BCL2 associated agonist of cell death (Bad) is a key substrate of AKT. Non-phosphorylated Bad inactivates the key anti-apoptotic protein of Bcl-2 through conjugation with it. However, Bad can be phosphorylated by AKT and then releases the Bcl-2. Free Bcl-2 shows powerful antiapoptotic activity and thus inhibits the apoptosis pathway [40, 41]. In the present study, we found that treatment with the natural drug of osthole can increase the expression of PTEN and thus inhibits the phosphorylation of AKT and Bad in CD133 positive HCC cells. As a result, osthole decreased the free Bcl-2 and obviously promoted the mitochondrial apoptosis induced cisplatin.

## CONCLUSIONS

We demonstrated the effect of osthole on partially reversing the cisplatin resistance of CD133 positive HCC cells in vitro and in vivo. Combination treatment with osthole and cisplatin may represent a novel strategy for the treatment of HCC.

## MATERIALS AND METHODS

### Cell lines

The human HCC cell lines Huh7 and HepG2 were purchased from the Cell Bank of the Type Culture Collection of the Chinese Academy of Sciences (Shanghai, China). Cells were cultured in RPMI-1640 medium (Gibco, Carlsbad, CA, USA) supplemented with 10% fetal bovine serum (Gibco). The cells were cultured at 37°C in a humidified incubator with 5% CO_2_. To obtain the CD133^+^ and CD133^-^ Huh7 and HepG2 cells, the cultured cells were stained with anti-CD133-FITC antibody (Miltenyi Biotec, Germany) for 20 min at room temperature. The population of CD133^+^ and CD133^-^ Huh7 and HepG2 cells were analyzed and sorted by using the fluorescent-activated cell sorting equipment (Beckman Coulter, USA).

### Gain-of-function and Loss-of-function of PTEN

To knockdown the gene of phosphatase and tensin homologue (PTEN), PTEN small interfering RNA (PTEN siRNA, Santa Cruz Biotechnology, Santa Cruz, CA, USA) was used. To overexpress PTEN, the PTEN eukaryotic expression plasmid was generated by cloning the open reading frame of the PTEN gene into the pcDNA3.1 plasmid (Life Technologies, Carlsbad, CA, USA). For transfection, cells were plated at 30-50% confluence. 24 h later, 50 pmol/ml RNA oligonucleotides or 2 μg/mL plasmids were transfected by using the Lipofectamine™ 2000 reagent (Invitrogen, Carlsbad, CA, USA) according to the manufacturer’s instruction.

### Quantitative real-time polymerase chain reaction (qRT-PCR)

Total RNA was extracted from cell lines by using Trizol reagent (Thermo Fisher Scientific, Inc., Waltham, MA, USA). cDNA was synthesized by using M-MLV Reverse Transcriptase (Thermo Fisher Scientific, Inc.) following the manufacturer's instruction. Polymerase chain reaction was performed by using a standard protocol from the SYBR Green PCR kit (TaKaRa, Dalian, China). GAPDH gene was used as the internal reference to determine the relative expression of PTEN through the 2^-ΔΔCT^ method.

### Cell viability assay

Transfected cells were seeded into 96-well culture plates at a density of 5,000 cells/well overnight. Cells were then treated with osthole (10 μmol/L) (Sigma-Aldrich, St. Louis, MO, USA) and different concentrations of cisplatin (0~30 μmol/L) (Sigma-Aldrich) for 48 h. Subsequently, CCK-8 (10 μl) (Beyotime, Shanghai, China) was added to each well and incubated for 2 h at 37°C. The absorbance of the plates was measured at 450 nm by using a microplate reader (Bio-Tek Instruments, Inc., Norcross, GA, USA). Half maximal inhibitory concentration (IC50) of cisplatin was calculated according to the cell viability curve. Combination index (CI) with cisplatin and osthole was calculated via the following formula: CI=E(A+B)/(EA+EB-EA×EB). EA represents as the inhibitory rate caused by cisplatin; EB represents as the inhibitory rate caused by osthole; E(A+B) represents as the inhibitory rate caused by Combination treatment with cisplatin and osthole. It is considered as simple addition of the two drugs when CI ranges from 0.85 to 1.15; It is considered as simple addition of the two drugs when CI ranges from 0.85 to 1.15; It is considered as the synergistic effect of the two drugs when CI is greater than 1.15; It is considered as the antagonistic effect of the two drugs when CI is less than 0.85.

### Immunoprecipitation

Cells were lysed in NP-40 buffer (Beyotime) and centrifuged at 12000g for 10 min. The resulting supernatants were incubated with primary antibody of Bad (Santa Cruz) overnight at 4 °C. Subsequently, supernatants were incubated with Protein A/G PLUS-Agarose (Santa Cruz) for 2 h. Next, the resulting supernatants were washed with cold NP-40 buffer. The co-precipitated proteins were removed from the agarose beads by boiling in sodium dodecyl sulfate (SDS) sample buffer.

### Western blot analysis

Total protein was extracted from cell samples by using RIPA buffer (Beyotime). 50 μg of the extracted and the co-precipitated proteins were separated by 10 % sodium dodecyl sulfate polyacrylamide gel electrophoresis (SDS-PAGE) and transferred to a PVDF membrane (Millipore, Billerica, MA, USA). After blocking in 5% nonfat milk for 2 h at room temperature, the membranes were incubated with anti-p-Bad (1:200, Santa Cruz), anti-p-AKT (1:200, Santa Cruz), anti-PTEN (1:200, Santa Cruz), anti-Bad (1:200, Santa Cruz), anti-AKT (1:200, Santa Cruz), anti-Bcl-2 (1:200, Santa Cruz), anti-cytochrome c (1:200, Santa Cruz), anti-caspase-9 (1:200, Santa Cruz) and anti-caspase-3 (1:200, Santa Cruz). After incubation with primary antibodies, membranes were washed and incubated with a horseradish peroxidase-conjugated secondary antibody (Santa Cruz) for 2 h at room temperature. Proteins on the membrane were visualized by using an enhanced chemiluminescence detection kit (Pierce, Rockford, IL, USA). Glyceraldehyde-3-phosphate (GAPDH) was used as an internal control to ensure equal protein loading. Mitochondria/Cytosol Fraction Kit (BioVision, Milpitas, CA, USA) was used to separate the mitochondria fraction and cytosol fraction before detection of cytochrome c.

### Mitochondrial membrane potential (ΔΨ_m_) and cell apoptosis

For detection of mitochondrial membrane potential (ΔΨ_m_), cells were collected and washed with PBS. Subsequently, cells were stained with 5,5′,6,6′-tetrachloro-1,1′,3,3′-tetraethyl imidacarbo cyanine iodide (JC-1, Molecular Probes, Carlsbad, CA, USA) in a 5% CO_2_ incubator at 37 °C for 20 min away from light. The samples were then analyzed by flow cytometry. Cells emitting red fluorescence were considered as cells with high ΔΨ_m_. For measurement of cell apoptotic rate, cells were collected and washed with PBS. Subsequently, Annexin V-FITC Apoptosis Detection Kit (Sigma-Aldrich) was used to measure the apoptotic rate.

### In vivo experiment

CD133 positive Huh7 cells were inoculated subcutaneously into the BALB/c nude mice (Shanghai Super-B&K Laboratory Animal Corp., Ltd., Shanghai, China). Cisplatin (8 mg/kg) and osthole (20 mg/kg) were administrated by intraperitoneal injection twice a week after xenografts reached 0.5 cm in diameter. Tumor size was measured every three days. Animals were killed 28 days post-injection. The animal care and experimental protocols were approved by the Animal Care Committee of The First Hospital, Jilin University.

### Statistical analysis

All data are represented as the mean ± standard deviation (SD) and carried out by at least three independent experiments. Differences between two groups were analyzed by two-tailed Student’s *t*-tests. Differences among multiple groups were analyzed by one-way analysis of variance and Bonferroni’s *post hoc* test. Statistical analysis was performed by using SPSS 15.0 software (SPSS Inc., Chicago, IL, USA). *P* < 0.05 was considered to be statistically significant.
